RETRACTED

# Exploring the potential effect of COVID-19 on an endangered great ape

**DOI:** 10.1038/s41598-021-00061-8

**Published:** 2021-10-21

**Authors:** Fernando Colchero, Winnie Eckardt, Tara Stoinski

**Affiliations:** 1 Department of Mathematics and Computer Science, University of Southern Denmark, Campusvej 55, 5230 Odense, Denmark; 2 Interdisciplinary Center on Population Dynamics, University of Southern Denmark, Campusvej 55, 5230 Odense, Denmark; 3 The Dian Fossey Gorilla Fund, 800 Cherokee Ave SE, Atlanta, GA 30315 USA

**Keywords:** Ecological modelling, Viral infection, Population dynamics

## Abstract

The current COVID-19 pandemic has created unmeasurable damages to society at a global level, from the irreplaceable loss of life, to the massive economic losses. In addition, the disease threatens further biodiversity loss. Due to their shared physiology with humans, primates, and particularly great apes, are susceptible to the disease. However, it is still uncertain how their populations would respond in case of infection. Here, we combine stochastic population and epidemiological models to simulate the range of potential effects of COVID-19 on the probability of extinction of mountain gorillas. We find that extinction is sharply driven by increases in the basic reproductive number and that the probability of extinction is greatly exacerbated if the immunity lasts less than 6 months. These results stress the need to limit exposure of the mountain gorilla population, the park personnel and visitors, as well as the potential of vaccination campaigns to extend the immunity duration.

## Introduction

Understanding the factors that influence the population dynamics of endangered species is fundamental for implementing successful management and conservation plans^1^. Diseases can be among the most important drivers of fluctuations in the demography and dynamics of wild populations, particularly for highly social species such as primates^2^. For instance, Ebola outbreaks have been linked to massive die offs of western lowland gorillas (*Gorilla gorilla*) and chimpanzees (*Pan troglodytes*) in Gabon and Congo, where over 3500 gorillas were suspected to have died of the disease between 2003 and 2004^3,4^.

Among primates, and in particular for great apes, there is a constant risk of disease transmission from humans because of their close genetic relatedness^5–8^ (for an overview see Gilardi et al*.*^9^). For example, severe respiratory disease outbreaks among chimpanzees in Côte d’Ivoire, Uganda and Tanzania, and mountain gorillas (*Gorilla beringei*) in Rwanda have been linked to human-born viruses^10–13^, while polio-like outbreaks of likely human origin have been recorded within chimpanzee populations in Tanzania and the Democratic Republic of the Congo^14^. This potential risk of transmission from humans to wildlife makes emergent diseases such as COVID-19 specially alarming due to the lack of knowledge of their short- and long-term impact on wild ape populations. To discover the severity and long-term implications of particular diseases on population persistence, it is crucial to anticipate the potential impact of emergent diseases such as COVID-19 on the dynamics of small populations of endangered primates, by means of predictive epidemiological and demographic models.

RETRACTED

Mountain gorillas (*Gorilla beringei beringei*), classified as endangered by the International Union for the Conservation of Nature (IUCN) Red List, have been the focus of intense study on the potential effects of diseases, particularly given that a significant percentage of the population is habituated and in close contact with humans on a daily basis for ecotourism, protection and research programs^12,15,16^. Respiratory outbreaks occur on almost an annual basis—between 1990 and 2020, 18 outbreaks were recorded in the groups within Volcanoes National Park^17^—and pneumonia is considered the second highest cause of mortality, although in only a few cases have illness be directly linked to human origins due to limited molecular data^12,18^. In 1988 an outbreak of respiratory illness in the Volcanoes National Park was linked to measles as the probable primary cause of infection, most likely transmitted from humans^19,20^. Importantly, to prevent further measles cases, a vaccination campaign was carried out after which no new cases were recorded.

The COVID-19 pandemic, produced by the sever acute respiratory syndrome coronavirus 2 (SARS-CoV-2) has resulted in an unprecedented worldwide economic, social and health crisis. Among humans, SARS-CoV-2 is spread primarily via respiratory droplets, with an average time from exposure to onset (i.e. serial interval) between 4.2 and 7.5 days and a mean incubation period between 4.8 and 9 days^21^. The virus can be spread by asymptomatic and symptomatic carriers and acute symptoms result in hospitalisations due to pneumonia and multiorgan diseases^22^. The basic reproductive number (*R*_0_), which corresponds to the average number of infections generated by one case, has been estimated to vary between 1.5 and 6.5 depending on the region and method of estimation^23^. The severity of the disease has been found to change with the age of the carrier, whereby older individuals are at a higher risk of developing acute symptoms, which also results in increased infection fatality rate with increasing age^22,24,25^.

RETRACTED

Recent research has found that great apes have the same cellular receptor protein for COVID-19 virus, SARS-CoV-2, as humans^26^. The susceptibility of gorillas was recently confirmed after a group of western lowland gorillas at the San Diego Wild Animal Park were diagnosed with COVID-19^27,28^. All individuals within the group were suspected to have contracted the virus and, although most individuals showed mild symptoms, pneumonia was diagnosed in a 48-year-old male, who recovered after being treated with steroids, antibiotics, and monoclonal antibodies—a regimen that would not be possible for wild ape populations. While overall this is positive news, the fact that 100% of the group became infected and 12% showed severe symptoms underscores the potential risk of COVID-19 to wild apes, particularly those with small population sizes living at high population densities in close proximity to humans—a situation that describes the two remaining populations of mountain gorillas.

Simulation models have been developed to explore the potential impact of infectious diseases in a population, particularly in the absence of accurate epidemiological data or to determine public health interventions to attenuate their effects^28–31^. Among the most used models are the Susceptible-Infected-Recovered (SIR) discrete time models^32^, which have been extended to account for the age-structure of the population^31^. Extensions of the SIR allow to include additional stages such as the SIRS model that assumes that recovered individuals may not maintain immunity, or the SIADE model that incorporates public health strategies such as self-isolation into the model^33^.

To evaluate the effect of COVID-19 on the mountain gorilla population dynamics, we constructed simulation models that combined population dynamics and epidemiological models, these last using its effect on humans as a benchmark. We used these models to measure the sensitivity of different measures of population performance to variations of four determinant aspects of the dynamics of the disease: (a) the basic reproductive number (*R*_0_), which measures the average number of future infections per newly infected individual when all individuals start as susceptible; (b) the infection fatality rate, which measures the probability of dying given that the individual has been infected; (c) the probability of becoming immune; and (d) the duration of immunity. The large body of research accumulated in the last year on the COVID-19 pandemic provides estimates for all four variables on humans (see “Materials and methods”), enabling us to incorporate epidemiological models such as SIRS into a fully age-sex-dependent stochastic population model. We parameterized several of the epidemiological variables in the SIR model based on recent results on humans and, since the extent by which gorillas would respond similarly to humans is unclear, we varied the values for these variables (R_0_, infection fatality rate, probability and duration of immunity) to run sensitivity analyses on the role that each of these played on the short and long-term chances of the population to survive.

RETRACTED

## Results

To predict the potential impact of COVID-19 on population dynamics, we combined an age- and sex-dependent stochastic population model with a fully sex-age-dependent SIRS model (Figs. 1 and 2). Because there are no known outbreaks of COVID-19 among populations of mountain gorillas, we used published information on the pandemic among humans for four epidemiological variables, namely (a) the basic reproductive number (*R*_0_)^34,35^, (b) the infection fatality rate (IFR)^24,25,36,37^, (c) the probability of developing immunity and (d) the duration of immunity^37–41^. We adjusted both, the infection fatality rate and the immunity probability to the lifespan of the gorillas by means of logistic functions of age (Fig. 2). To account for the lack of epidemiological information in mountain gorillas, we tested a range of scenarios in which we used different values for each of these epidemiological variables. Specifically, we varied *R*_0_ between 0.5 and 6, the immunity duration, *T*_*I*_, between 1 and 12 months, the maximum infection fatality rate, *q*_*M*_, between 0.3 and 0.6, and the maximum immunity probability, *M*_*I*_, between 0.2 and 0.8, for a total of 800 scenarios (for further details see “Materials and methods”). For each scenario, we ran 2000 stochastic simulations each starting with a single infected individual.

**Figure 1:** Conceptual epidemiological model applied to the study subpopulation. The time units are half months, and each stage (susceptible, infected, immune, dead) is fully age-dependent. The background mortality follows the sex-age-specific mortality estimated on the last 40 years of demographic information of the study population.

**Figure 2:** Age-specific infection fatality rate (IFR) (**A**) and immunity probability (**B**) used to model the potential impact of COVID-19 on the dynamics of the study population. The color gradient is only used to stress the gradual nature of the values.

Our simulations showed that the most important epidemiological variable on the reduction in the study subpopulation during the first 2 years of simulation was the basic reproductive number, *R*_0_, where, in most cases, the population declined for *R*_0_ values equal or larger than 1.05 (Figs. 3 and 4). Only when the immunity duration was of 12 months population declines were delayed until *R*_0_ reached higher values (e.g. 1.3). However, as expected, the decline was steeper for all scenarios for the higher maximum infected mortality, *q*_*M*_, of 0.6. In those cases, the populations could decline by up to 40% for an immunity duration of 1 or 3 months and a *R*_0_ of 6, irrespective of the maximum immunity probability, *M*_*I*_. The maximum immunity probability, *M*_*I*_, only made a difference when the immunity duration was of 6 or 12 months. In these cases, higher immunity duration was associated with lower population decline.

RETRACTED

**Figure 3:** Change in the size of the study population 2 years after the initial infection as a function of COVID-19 epidemiological variables, namely, the maximum infection fatality rate (*q*_*M*_), the basic reproductive number (*R*_0_), the maximum immunity probability (*P*_*I*_), and the immunity duration in months (*T*_*I*_).

**Figure 4:** Percent increase or decline in the population as a function of the disease’s basic reproductive number (*R*_0_) between the first and second years after the initial infection. The colored lines show four different levels of maximum immunity probability (i.e. *P*_*I*_ of 0.2, 0.4, 0.6, 0.8). The horizontal grey lines show the level at which the population is stationary, and the vertical dashed lines show the mean human *R*_0_.

To understand the long-term impact of a disease outbreak in the study population, we ran additional simulations for 50 years for the scenarios with an immunity duration, *T*_*I*_, of 3 and 12 months and a maximum immunity probability, *M*_*I*_, of 0.2. Here, we found that, in the absence of new external infections and if the disease did not drive the population to extinction, then the disease would eventually disappear from the subpopulation, on average, after 10–16 years (Fig. 5). Interestingly, for the scenario with an immunity duration of 12 months and a maximum infection mortality probability of 0.3, the disease took longest to disappear (i.e., 16 years). However, the proportion of extinct subpopulations for all scenarios was considerably high (Fig. 6), particularly when the immunity duration lasted only 3 months and the maximum infected mortality probability was 0.6. In that case, close to 80% of the subpopulations went extinct after 50 years.

**Figure 5:** Average predicted long-term effect of COVID-19 on the Karisoke mountain gorilla subpopulation when the basic reproductive number is *R*_0_ = 3 and the maximum immunity probability is *M*_*I*_ = 0.2 for four scenarios resulting from the combination of an immunity duration (*T*_*I*_) of 3 or 12 months and maximum infected mortality probability (*q*_*M*_) of 0.3 or 0.6.

RETRACTED

**Figure 6:** Cumulative number of extinct subpopulations as a function of time based on the simulated effect of COVID-19 on the study mountain gorilla population. These simulations correspond to a basic reproductive number of *R*_0_ = 3 and a maximum immunity probability is *M*_*I*_ = 0.2 for four scenarios resulting from the combination of an immunity duration (*T*_*I*_) of 3 or 12 months and maximum infected mortality probability (*q*_*M*_) of 0.3 or 0.6.

## Discussion

In the case of a potential outbreak of COVID-19 in the Karisoke mountain gorilla subpopulation, our simulations provided key insights into the influence of several of the epidemiological variables associated to the disease. We found that the basic reproductive number, *R*_0_, played a crucial role in the chances of extinction of the subpopulation, where values higher or equal to 1.05 would drive the population to decline and therefore increasing dramatically its probability of going extinct. Notably, the average *R*_0_ in humans has been estimated at around 2.5 new cases per infected individual, with reported values ranging from 1.5 to over 7 depending on the estimation method and on the population studied^34^. However, due to the group dynamics of gorilla populations, whereby groups are not constantly in contact, it is likely that *R*_0_ is lower in this species. However, it is probable that *R*_0_ will be strongly influenced by group density and the overall social structure or the population (e.g. few large groups versus many small groups within the same space)^42^, which is why we modeled a range of *R*_0_ values. For example, increased group density is associated with increased intergroup interactions^42,43^, which presumably would enhance the opportunity for COVID-19 to pass from one group to another, thus increasing *R*_0_. The potential transmission of diseases like COVID-19 between social groups is an important area of future study (for respiratory diseases on this population see^44^. Nonetheless, our finding that there is a threshold value of *R*_0_ = 1.05 above which the subpopulations start declining highlights the current risk of an outbreak on the subpopulation.

Importantly, we found that, at similar values of the COVID-19 epidemiological variables (i.e., R0 ≈ 2.5–3, *q*_*M*_ = 0.3, *T*_*I*_ = 3 months, and *M*_*I*_ = 0.2) to those reported for humans, up to 71% of the long-term simulated subpopulations went extinct after 50 years. However, due to the availability of health care among humans, it is likely that the maximum infected mortality probability among humans (*q*_*M*_ = 0.3) would be an under-estimate for gorillas. Therefore, it is important to consider for any prevention plan the results from our long-term simulations using a higher value of *q*_*M*_ = 0.6, which yielded an even higher risk of extinction of close to 80% of the simulated subpopulations. Interestingly, the simulations showed that, if the subpopulations did not go extinct and were not exposed to new external infections, the disease eventually disappeared after an average maximum of 16 years.

RETRACTED

Our results support management and best practices recommendations as those provided by the Section of Great Apes of the Primate Specialist Group of the IUCN Species Survival Commission^45^. The most evident and urgent goal is to avoid infection with COVID-19. This requires that both, park personnel and tourists are vaccinated promptly, monitored for evidence of infection before they come in proximity of the mountain gorillas, and that mask wearing, hygiene measures and daily health checks before visiting gorillas are strictly followed. Similarly, it is fundamental to establish a monitoring protocol that allows testing regularly gorillas for possible infections. If individuals become infected, priorities should focus on avoiding any new external infections by following the recommendations above, and to keep *R*_0_ below 1. The latter could be potentially achieved through decreasing group density, for instance, controlling the movement of the groups so that inter-group interactions and close proximity are minimized. In addition, symptomatic individuals need to be closely monitored and their infection measured for instance, by collecting fecal samples that can be immediately analyzed, to accurately record the progression of the disease and implement disease spread prevention measures.

Extending the duration of immunity can importantly reduce the chances of extinction. The respiratory disease outbreak in 1988 attributed to measles that was seemingly controlled through a vaccination campaign provides a good model for the potential benefit of a COVID-19 vaccine protocol^19,46^. However, it is important to stress that such a vaccination campaign was possible in part because the gorillas were both habituated and observed daily, meaning that the disease was identified and veterinarians could vaccinate^19,46^. Therefore, this approach likely will only be possible for habituated individuals. But given that these are the most at risk of exposure to COVID-19, the feasibility of a vaccination campaign should be a priority.

In the longer term, minimizing *R*_0_ in mountain gorillas could involve decreasing the frequency of group interactions^44^, by minimizing any risk of human disturbance to existing habitat allowing groups to spread out to the maximum extent and also expanding the park.

RETRACTED

Although our results show that the measures we propose above are key to ensure the survival of the subpopulation, the most promising public health alternative is the one health approach^45–49^. The one health approach stresses the tight relationship between human, animal and environmental health, and that, ensuring health and well-being in humans requires an integrative approach that extends to ecosystem health. In the case of the risk of COVID-19 infection among gorillas and primates in general, this approach results into a two-way avenue. Namely, that transboundary public health efforts to control the disease among humans, especially those working in or visiting the park as well as local communities living adjacent to the park boundaries, would directly reduce the risk of infection among wild populations^49^.

## Materials and methods

### Study site and demographic data

The study was carried out in Volcanoes National Park, the Rwandan part of the Virunga massif, which is further shared with Uganda and the Democratic Republic of the Congo. We focused on habituated mountain gorilla groups monitored by the Dian Fossey Gorilla Fund’s Karisoke Research Center, often referred to as the Karisoke subpopulation. Since 1967, groups in this subpopulation have been followed on a near daily basis. Through the mid-2000s, the Karisoke groups generally numbered three but over the last decade, group fission events and new group formations resulted in an average of ten groups in the region (see^42,43^). During daily observations, detailed demographic data are recorded, such as group composition, birthdate and death date, group transfers (for further details see Strier et al.^50^). The data used for this study covers demographic data from 1967 to 2018 and includes 396 recognized individuals.

### Epidemiological data

We obtained published data on four variables that control the disease dynamics of COVID-19 in humans, namely (a) the basic reproductive number (*R*_0_)^34,35^, (b) the infection fatality rate (IFR) based on estimates from China and Italy^24,25,36,37^, (c) the probability of developing immunity and (d) the duration of immunity^37–41^.

### Stochastic projection model

We used the stochastic projection model proposed by Colchero et al*.*^51^, that models population dynamics for both sexes on fully age-dependent demographic rates. The model incorporates the yearly variance–covariance between demographic rates, while it accounts for infanticide as a function of the number of silverbacks (mature males > 12 years old) in the population^51^. Because of this relationship between infanticide and number of silverbacks, this source of mortality changes in time and cannot be assumed to be part of the infant mortality rate. To explore the extinction probability for the Karisoke subpopulation as a function of different diseases, we gathered information from the model on the proportion of individuals that died for each disease and the frequency of outbreaks (i.e., how often outbreaks occurred).

RETRACTED

### Demographic-epidemiological projection model for COVID-19

We constructed a predictive population model that combines the species’ baseline demographic rates with a model based on the susceptible-infected-recovered-susceptible (SIRS) framework. As the baseline demographic rates, we used the age-specific mortality and fecundity estimated by Colchero et al.^51^ for mountain gorillas (Karisoke subpopulation). We defined four epidemiological stages, namely (a) susceptible, (b) infected, (c) immune and (d) dead, each of which we further divided into a fully age-specific structure (Fig. 1). Based on recent research on COVID-19 on humans, we assumed that the dynamics of the model allowed for the recovered individuals to be divided into either susceptible or immune^37–41^. Furthermore, we incorporated the potential age-specific infection fatality rate (IFR) based on current estimates from medical and epidemiological research^24,25,36,37^, adjusted to the lifespan of the gorillas by means of the logistic function

1 $$q\left(x\right)=\frac{{q}_{M}}{1+{\text{exp}}\left[-0.2\left(x-25\right)\right]},$$

where *q*_*M*_ is the maximum infected mortality probability. Similarly, we modeled the probability of developing immunity as a function of the strength of the disease, which, based on recent research, we measured as mirroring Eq. (1) as

2 $$m\left(x\right)=\frac{{M}_{I}}{1+{\text{exp}}\left[-0.2\left(x-25\right)\right]},$$

where *M*_*I*_ is the maximum immunity probability (Fig. 2B).

To explore the potential impact of COVID-19 on the growth rate of the Karisoke mountain gorilla subpopulation, we varied four of the critical epidemiological variables, namely (a) the basic reproductive number, *R*_0_, from 0.5 to 6 (which helps to simulate factors such as increased group density, which may increase the likelihood of transmission), (b) the maximum infected mortality probability, *q*_*M*_ = (0.3, 0.6) (Fig. 2A), (c) the immunity duration, *T*_*I*_ to 1, 3, 6, and 12 months, and (d) the maximum immunity probability, *M*_*I*_, from 0.2 to 0.8 (Fig. 2B). As time units we used year fractions in half months (i.e., *t*_1_ − *t*_0_ = 0.5/12), which allowed us to simplify the model, based on current information on the average time of serial interval and incubation period in humans^21^. This implementation assumes that susceptible individuals could become infected at the beginning of the time interval, while infected individuals in time interval *t* would either recover (immune or susceptible) or die in *t* + 1.

RETRACTED

The deterministic structure of the model implies that the number of individuals in each sex, age and epidemiological stage was given by the possible contribution from the other stages 1/2 month before. This is, the number of susceptible individuals of age *x* at time *t* is given by the difference equation

$$\begin{aligned} n_{s,x,t} & = p_{x - 1} \left\{ {n_{s,x - 1,t - 1} + n_{i,x - 1,t - 1} \left[ {1 - q\left( {x - 1} \right)} \right]\left[ {1 - m\left( {x - 1} \right)} \right]} \right\} \\ & \quad + n_{{m,x - T_{i} ,t - T_{i} }} \prod\limits_{{j = x - T_{i} :j > 0}}^{x - 1} {p_{j} - n_{i,x,t} } , \\ \end{aligned}$$

where the *n*_*s,x,t*_ is the number of susceptible individuals of age *x* at time *t*, and subscripts *i* and *m* refer to infected and immune individuals, respectively. For simplicity of notation, we do not include a subscript for sex, although the model does distinguish between sexes. The probability *p*_*x*_ is the age-specific survival probability. Functions *q*(*x*) and *m*(*x*) are as in Eqs. (1) and (2). Similarly, the number of immune individuals at time *t* and age *x* are

$${n}_{m,x,t}={n}_{i,x-1,t-1}\left[1-q\left(x-1\right)\right]m\left(x\right)+\sum_{\{j:0\le j\le {T}_{i}\wedge x-j>0\}}{p}_{x-j}{n}_{i,x-j,t-j}.$$

We incorporated this mechanistic structure into a stochastic model, where all contributions from time *t* to *t* + 1 were drawn from binomial or Poisson distributions. For instance, the total new number of infected individuals, *N*_*i,t*_, was obtained as a random draw from a Poisson distribution with expected value

$$E\left[{N}_{i,t}\right]={\text{min}}\left[{{R}_{0}N}_{i,t-1},{N}_{t}\right],$$

where *N*_*t*_ is the total number of individuals in the study subpopulation. We then distributed randomly these individuals into different available ages and sex corresponding to the term *n*_*i,x,t*_, in the susceptible equation above. The number of newborns, *B*_*x,t*_, at each age for which there were available females at time *t* was drawn from a binomial distribution with expected value

$$E\left[{B}_{x,t}\right]=\left({n}_{s,x,t}+{n}_{m,x,t}\right){f}_{x}$$

where *f*_*x*_ is the age-specific average female fecundity rate and *n*_*s,x,t*_ and *n*_*m,x,t*_ refers to the number of susceptible and immune females, respectively, of age *x* at time *t*. The sex of each newborn was then determined by means of a Bernoulli draw with probability given by the proportion of males in the population. Thus, if the draw produced 1 for that individual, it became a male, and if 0 a female.

RETRACTED

For each scenario, we ran stochastic simulations for 2000 iterations for 10 years and recorded the average number of individuals at each age–sex and epidemiological state at every month. We then ran long-term stochastic simulations for four scenarios with *R*_0_ = 3 and maximum immunity probability *M*_*I*_ = 0.2. For these, we recorded also the number of subpopulations that went extinct at each month.

## Data Availability

Computer code and tutorial can be found at https://github.com/fercol/popDisease.
